# Silencing circular RNA VANGL1 inhibits progression of bladder cancer by regulating miR‐1184/IGFBP2 axis

**DOI:** 10.1002/cam4.2650

**Published:** 2019-11-23

**Authors:** Dengke Yang, Haining Qian, Zhen Fang, An Xu, Shutian Zhao, Bingyan Liu, Dong Li

**Affiliations:** ^1^ Department of Urinary Surgery Tongren Hospital Shanghai Jiaotong University School of Medicine Shanghai China; ^2^ Department of Interventional Radiology Tongren Hospital Shanghai Jiaotong University School of Medicine Shanghai China

**Keywords:** metastasis, microenvironment, signal transduction

## Abstract

Circular RNA VANGL1 (circVANGL1) is generated from two exons of the Van Gogh‐like 1 (VANGL1) gene and serves as a tumor promoter by sponging certain microRNAs (miRNAs). However, the role of circVANGL1 in bladder cancer (BC) is still unclear. So, in order to investigate the role of circVANGL1 in BC, quantitative reverse transcription‐polymerase chain reaction (qRT‐PCR) was employed to evaluate the circVANGL1 expression in tumor tissues from BC patients and in BC cell lines. Small interfering RNA against circVANGL1 was constructed and stably transfected into human bladder epithelium immortalized cells (SV‐HUC). Cell invasion and migration were detected in Transwell chambers, cell proliferation was determined by CCK8 assays, and tumorigenesis in nude mice was examined to assess the effect of circVANGL1 in BC. Subcellular localization of circVANGL1 was confirmed by fluorescence in situ hybridization. The interactive relationships among circVANGL1, miRNA, and relative proteins were confirmed by luciferase reporter assays. The results showed that circVANGL1 was upregulated in both BC tissues and cell lines. Silencing the expression of circVANGL1 suppressed cell invasion, migration, and proliferation during in vitro experiments. Mechanistically, we demonstrated that circVANGL1 upregulated the expression of miR‐1184 target gene insulin‐like growth factor‐binding protein 2 (IGFBP2) by sponging miR‐1184, which promoted the aggressive biological behaviors of BC. Taken together, our results indicate that circVANGL1 acts as a tumor promoter through the novel circVANGL1/miR‐1184/IGFBP2 axis. Hopefully, our study will provide new ideas for the clinical treatment of BC.

## Graphical abstract

Circular RNA VANGL1 (circVANGL1) upregulated the expression of miR‐1184 target gene insulin‐like growth factor‐binding protein 2 (IGFBP2) by sponging miR‐1184, which promoted the aggressive biological behaviors of BC. Taken together, our results indicate that circVANGL1 acts as a tumor promoter through the novel circVANGL1/miR‐1184/IGFBP2 axis.

## 1 INTRODUCTION

Bladder cancer (BC) is among the most popular urinary system disease in the world, which causes estimated 165 000 deaths and 429 000 new cases each year.^1^, ^2^ Despite new promising treatments, BC recurrence rate within 5 years remains significant (15%‐90%),^3^, ^4^, ^5^, ^6^ and long‐term clinical treatment brings heavy economic burdens to both patients and society.^7^ So it is crucial to find novel diagnostic and therapeutic BC targets.

Circular RNA (circRNA) is a class of endogenous noncoding RNAs constructed by a closed circular structure.^8^, ^9^ Previous investigations have revealed that circRNAs differential expression is tightly associated with cancer progression.^10^ These data also suggested that circRNAs abnormal expression is related to BC progression. For example, circPTK2 expression upregulation promotes migration and proliferation of BC cells.^11^ More evidence informs that circRNAs function vitally in the regulation of gene expression. In one study, the aberrant expression of circRNA MYLK promoted BC progression by modulating the VEGFR2/VEGFA signaling pathway.^12^ Furthermore, the circRNA ITCH inhibited BC progression by sponging miR‐224/miR‐17 and regulating PTEN and p21 expressions.^13^ Previous studies found a series of differences and characterizations in circRNA expression profiles between bladder carcinoma tissues and adjacent noncarcinoma tissues using high‐throughput microarray assay. We reanalyzed the 20 upregulated and downregulated circRNAs found that circRNA VANGL1 (circVANGL1) (hsa_circ_0002623) also displays aberrant expression in BC, but whether circVANGL1 functions in BC progression is still unknown.^14^

As a group of tiny regulatory noncoding RNAs that conserved evolutionarily, microRNAs (miRNAs) have been advised to participate in the regulation of vary biological functions.^15^ By acting as sponges of miRNA, circRNAs can regulate gene expression by suppressing miRNA activity.^16^ However, the regulatory roles of circVANGL1 acting as a miRNA sponge in BC remain unclear.

The current research aim to detect circVANGL1 expression in BC and assess its biological mechanisms. Data illustrated that circVANGL1 was upregulated in BC and promoted cell migration and proliferation. The results thus point in new directions for the improvement of novel therapeutic processes toward BC in the clinic.

## 2 MATERIALS AND METHODS

### 2.1 Animal ethics statement

BALB/c nude mice (n = 12) that were 4 weeks old and weighted 15‐20 g (SLARC Inc) were utilized in this investigation. The Ethics Committee of Tongren Hospital‐affiliated Shanghai Jiaotong University School of Medicine approved the animal experiment.

### 2.2 Clinical tissue samples and ethics statement

Bladder cancer tumor and corresponding paracancerous tissue were extracted from patients who diagnosed with BC and had received surgery in the Tongren Hospital of Shanghai Jiaotong University School of Medicine between 2015 and 2017. Sixty pairs of tissues were frozen freshly and stored in liquid nitrogen. The Ethics Committee of Tongren Hospital‐affiliated Shanghai Jiaotong University School of Medicine approved the tissues used in this study for use.

### 2.3 Fluorescence in situ hybridization

Particular probes for the circVANGL1 sequence were employed for in situ hybridization, which was formerly provided as well.^17^ In sum, we utilized the probes that labeled with cy5 and 4,6‐diamidino‐2‐phenylindole as a cell nucleus counterstain. We performed all procedures according to the standard process (Genepharma).

### 2.4 circRNA analysis and target prediction

The hsa_circ_0002623 and miRNA target gene was predicted through the web‐based package ‘Circular RNA Interactome’.

### 2.5 Bifluorescein reporting experiment

We cotransfected HEK293T cells with miRNA mimics and with either plasmids containing mutant or wild‐type 3′‐UTR fragments from the gene for insulin‐like growth factor‐binding protein 2 (IGFBP2), or with the predicted binding sequence from circVANGL1, through Lipofectamine 2000 (Invitrogen). At 48‐hour posttransfection, a dual luciferase reporter assay system (Promega) was employed to detected renilla and firefly luciferase activities. Then the rates of luminescence between firefly and renilla luciferase were computed and every assay was replicated at least three times.

### 2.6 Cell culture

The human bladder epithelium immortalized cells (SV‐HUC) line and BC cell lines (T24, EJ, J82, RT‐4, UM‐UC‐3, and TCC) were supplied by the Type Culture Collection Affiliated to the Chinese Academy of Sciences (Shanghai, China) and cultivated under 37°C with 5% CO_2_ in dulbecco's modified eagle medium (DMEM) (Gibco), which contained 10% fetal bovine serum (Gibco).

### 2.7 Cell transfection

For miR‐1184 overexpression, we transfected UM‐UC‐3 cells with 50 nmol/L miR‐1184 mimics or negative control RNA (miR‐NC; GenePharma) via Lipofectamine 2000 and cultured them for 2 days (48 hours) before miR‐1184 expression analysis as well as further experiments. For miR‐1184 inhibition experiments, UM‐UC‐3 cells were pretreated with miR‐1184 inhibitor for 48 hours in prior performing miR‐1184 expression analysis and further experiments. For circRNA VANGL1 expression analysis, small interfering RNA (siRNA) over circRNA VANGL1 and a circRNA VANGL1 overexpression vector were constructed by GenePharma and transfected into UM‐UC‐3 cells at 50 nmol/L via Lipofectamine 2000. To achieve IGFBP‐2 overexpression, an IGFBP‐2 overexpression vector was performed by GenePharma. We transfected UM‐UC‐3 cells with either the IGFBP‐2 overexpression vector or a negative control at a concentration of 50 nmol/L through Lipofectamine 2000 following the manufacturer's process.

### 2.8 Cell viability assays

We analyzed cell viability by Cell counting kit‐8 (CCK8; Gibco). Briefly, we seeded 1 × 10^4^ UM‐UC‐3 cells into plates with 96 wells and incubated them over the night. Then we removed medium and washed cells with phosphate buffer solution (PBS) for three times. We added a mixture of 90 µL DMEM and 10 µL CCK8 to every well and incubated it under 37°C for 1.5 hours before optical density measurement at 450 nm.

### 2.9 Western blots

We extracted protein from cells through RIPA lysis buffer containing protease inhibitor (Sigma‐Aldrich) and measured the concentration with bicinchoninic acid (BCA) protein assay kits (Vigorous Biotechnology Beijing). Samples of 20‐μg protein were resolved using sodium dodecyl sulfate polyacrylamide gel electrophoresis (SDS‐PAGE) and transferred onto nitrocellulose membranes (Millipore). We blocked membranes with 5% nonfat dry milk for 2 hours before their incubation with primary antibodies under 4°C overnight. We used reduced glyceraldehyde‐phosphate dehydrogenase as the internal control. We incubated membranes with horseradish peroxidase‐coupled secondary antibodies for 1 hour under the room temperature.

### 2.10 Transwell assays

Invasion and migration were evaluated with Transwell chambers (Corning Life Sciences) using Matrigel (BD Biosciences), which was reported before.^18^ We stained cells with Crystal Violet of 0.1% and photographed them. The mean count of invasive or migratory cells was set as a percentage relative to controls. Results were based on three replicated experiments.

### 2.11 Wound‐healing assay

We seeded UM‐UC‐3 cells (5 × 10^5^) into plates with six wells and cultured them with DMEM. When cell confluency reached 90%, the culture medium was replaced with serum‐free DMEM. We used a pipette tip of 10‐µL to scratch a line and washed off the cast‐off cells with PBS. Migrating cells were observed after incubation for 24 hours.

### 2.12 RNA extraction and quantitative reverse transcription PCR

We isolated RNA from UM‐UC‐3 cells and tumor tissue through TRIzol reagent (TaKaRa). We employed PrimeScript^™^ RT Master Mix kits (TaKaRa) for first‐strand cDNA synthesis and performed quantitative reverse transcription PCR (qRT‐PCR) with Power SYBR Green PCR Master Mix (Life Technology) and primers. We employed *GAPDH* to be internal control. We utilized $2^{-\Delta \Delta C_{t}}$ method for the analysis of gene expression. The primer sequences were as follows: circVANGL1, 5′‐CTACAGCCTGGGACACCTGAG‐3′ (sense), 5′‐CCTCTGCCGTCTTTATTG‐3′ (antisense); IGFBP2, 5′‐ATGCTGCCGAGAGTGGGC‐3′ (sense), 5′‐CTACTGCATCCGCTGGGTG‐3′ (antisense); GAPDH, 5′‐GGTATCGTGGAAGGACTCATGAC‐3′ (sense), 5′‐ATGCCAGTGAGCTTCCCGT‐3′ (antisense).

### 2.13 Xenografts in mice

Totally, 5 × 10^6^ viable UM‐UC‐3 cells expressing wild‐type circVANGL1 or siRNA against circVANGL1 (sicircRNA) were injected into the right flanks of nude mice.^19^ Sizes of tumors were detected every 5 days via a Vernier caliper with tumor volume: 0.5 × length × width^2^. We euthanatized mice for qRT‐PCR analysis 30 days later from the implantation.

### 2.14 Statistics analysis

Data are denoted by means ± SD. GraphPad Prism (GraphPad) was utilized to compare differences between groups. *P* ≤ .05 indicated a statistical significance.

## 3 RESULTS

### 3.1 circVANGL1 expression is significantly increased in BC

Previous big data from microarray assays have found that circTCF25 overexpression promoted CDK6 expression by sponging miR‐103a‐3p and miR‐107, which eventually promoted BC cell migration and proliferation.^14^ In current research, the results of microarray assays illustrated that circVANGL1 (hsa_circ_0002623) was also expressed aberrantly. Circular RNA VANGL1 is derived from cyclizing two exons from the *VANGL1* gene. The spliced mature circRNA is 741 bp and *VANGL1* is 4628 bp, which is located at chr1: 116202261‐116206889 (Figure 1A). In order to investigate if circVANGL1 expression was changed in BC, 60 pairs of BC tissues and the adjacent normal tissues were studied via qRT‐PCR. Resulting data demonstrated that circVANGL1 expression in BC tissues increased comparing with matched adjacent normal tissues (Figure 1B). Also, circVANGL1 expression enhanced in 6 BC cell lines (J82, T24, EJ, RT‐4, UM‐UC‐3, and TCC) comparing with normal SV‐HUC urothelial cells. The output also illustrated that circVANGL1 expression was highest in UM‐UC‐3 cells comparing with other BC cell lines (Figure 1C). We thus chose UM‐UC‐3 cells to explore the circVANGL1 effect in fluorescence in situ hybridization assays, which demonstrated that circVANGL1 localized to the cytoplasm predominately (Figure 1D). In sum, these data advised that circVANGL1 may function importantly in the BC progression.

**Figure 1:** Circular RNA VANGL1 (circVANGL1) was significantly increased in bladder cancer (BC) and related BC cell lines. A, The genomic loci of the VANGL1 gene and circVANGL1. Green arrow indicates the back‐splicing. B, Quantitative reverse transcription PCR (qRT‐PCR) assays show circVANGL1 expression in BC tissues and corresponding adjacent normal tissues from 60 BC patients. Data are presented as means ± SD. ***P < .001 vs normal. C, qRT‐PCR assays show circVANGL1 expression in BC cell lines and SV‐HUC cells. Data are presented as means ± SD. **P < .01, ***P < .001 vs SV‐HUC cells. D, Fluorescence in situ hybridization was performed to determine the subcellular localization of circVANGL1. Scale bars: 10 μm

### 3.2 Silencing circVANGL1 in vitro inhibits BC cell invasion, migration and growth through inhibiting IGFBP‐2

To reveal the role of circVANGL1 in BC, sicircRNA was prepared and transfected into UM‐UC‐3 cells. Quantitative reverse transcription PCR detection suggested that circVANGL1 expression in UM‐UC‐3 cells was downregulated 48 hours post‐sicircRNA transfection compared with NC or nontransfected control cells (Figure 2A). Western blot experiments indicated that IGFBP2 expression was also decreased in UM‐UC‐3 cells after circVANGL1 was silenced, while cotransfection of the IGFBP2 overexpression vector restored and actually increased IGFBP2 expression compared with control or circVANGL1‐downregulated cells (Figure 2B,C). Insulin‐like growth factor‐binding protein 2, a key antiapoptotic regulator, as a molecular target of the PI3K/AKT/mTOR pathway.^20^ Moreover, several malignancies are characterized by increased IGFBP2 expression.^21^ Suggestion that IGFBP2 was the downstream target of circVANGL1. CCK8 assays showed that downregulating circVANGL1 expression decreased the UM‐UC‐3 cell proliferation significantly comparing with the control group; in contrast, IGFBP2 overexpression increased the UM‐UC‐3 cell proliferations even after downregulation of circVANGL1 (Figure 2D). Wound‐healing assays informed that circVANGL1 downregulation caused slower closure of scratch wounds comparing with the control group, while IGFBP2 upregulation promoted more rapid closing of scratch wounds (Figure 2E). Also, Transwell invasion and migration assays demonstrated that the invasive and migratory capacity of UM‐UC‐3 cells was diminished after silencing circVANGL1 but was restored after increasing IGFBP2 expression (Figure 2F‐H). The implication from these experiments was that silencing circVANGL1 inhibited BC cell migration, invasion and growth via downregulation of IGFBP‐2, although the exact mechanism remains unclear.

**Figure 2:** Silencing circular RNA VANGL1 (circVANGL1) inhibits bladder cancer (BC) cell growth, migration and invasion by inhibiting insulin‐like growth factor‐binding protein 2 (IGFBP‐2) in vitro. A, Quantitative reverse transcription PCR (qRT‐PCR) detection shows circVANGL1 expression after transfection with small interfering RNA (siRNA) against circVANGL1. Data are presented as means ± SD. ***P < .001 vs control. B, Western blots show IGFBP‐2 expression. C, Relative protein levels were analyzed and data are presented as means ± SD. ***P < .001 vs control. ^###^ *P* < .001 vs siRNA against circVANGL1 (sicircRNA). D, CCK8 assays were performed to assess cell proliferation. Data are presented as means ± SD. ***P < .001. E, Wound‐healing assays showed that circVANGL1 downregulation resulted in slower closure of scratch wounds. Scale bars: 50 μm. F‐H, Cell migration and invasion were determined in UM‐UC‐3 cells using transwell assays. Data are presented as means ± SD. ***P < .001 vs control. ^###^ *P* < .001 vs sicircRNA. Scale bars: 30 μm

### 3.3 Ectopic miR‐1184 expression suppresses UM‐UC‐3 cell migration, invasion and growth by targeting IGFBP‐2 gene

Bioinformatics analysis through ‘Circular RNA Interactome’ showed that miR‐1184 was a candidate circVANGL1 target. To identify a role for miR‐1184 in BC progression, we constructed a miR‐1184 overexpression vector and transfected it into UM‐UC‐3 cells. Quantitative reverse transcription PCR assays detected that miR‐1184 expression significantly increased after the miR‐1184 expression mimic compared with NC or control cells (Figure 3A). Western blotting showed that IGFBP2 expression was simultaneously reduced regarding UM‐UC‐3 cells with miR‐1184 upregulation. Furthermore, the loss of IGFBP2 expression caused by the miR‐1184 mimic was reversed by IGFBP2 overexpression even when the mimic was present (Figure 3B,C). CCK8 analysis then revealed that upregulating miR‐1184 expression decreased the UM‐UC‐3 cell proliferations significantly comparing with the control group, while overexpression of IGFBP2 increased the UM‐UC‐3 cell proliferation even after miR‐1184 upregulation (Figure 3D). Wound‐healing assays demonstrated that miR‐1184 upregulation caused slower closure of scratch wounds comparing with control cells, while upregulation of IGFBP2 promoted faster closure of scratch wounds comparing with the control group (Figure 3E). Finally, Transwell invasion and migration assays inferred that invasion and migration by UM‐UC‐3 cells decreased after stimulating miR‐1184 expression but increasing IGFBP2 expression reversed these effects (Figure 3F‐H). Our results thus suggest that overexpressing miR‐1184 inhibits BC cell growth, migration and invasion by downregulating IGFBP‐2.

**Figure 3:** Ectopic expression of miR‐1184 suppresses UM‐UC‐3 cell growth, migration and invasion by targeting the insulin‐like growth factor‐binding protein 2 (IGFBP‐2) gene. A, RT‐PCR assay shows miR‐1184 expression after transfection with miR‐1184 mimics. B, Western blot shows IGFBP‐2 expression. C, Relative protein levels were analyzed, and data are presented as means ± SD. ***P < .001 vs control. ^###^ *P* < .001 vs mimic. D, CCK8 assays were performed to assess cell proliferation. E, Wound‐healing assay showed that downregulating miR‐1184 resulted in faster closure of scratch wounds. Scale bars: 50 μm. F‐H, Cell migration and invasion were determined in UM‐UC‐3 cells using Transwell assays. Data are presented as means ± SD. ***P < .001 vs control. ^###^ *P* < .001 vs mimic. Scale bars: 30 μm. I, Binding sites of miR‐1184 in the 3′UTR of IGFBP‐2 were predicted. The mutated version of the IGFBP‐2 3′UTR is also shown. J, The relative luciferase activity was determined 48 h after transfection with miR‐1184 mimic/NC or with the 3′UTR of IGFBP‐2 wild type (WT)/Mutant (Mut) in HEK293T cells. Data are presented as means ± SD. ***P < .001 vs control

Analysis further verified that miR‐1184 can interact with the IGFBP2 3′UTR and suppress IGFBP2 expression via a posttranscriptional mechanism. Dual luciferase reporter assays were therefore conducted to validate this hypothesis. Wild‐type 3′UTR sequence from IGFBP2 gene and mutated 3′UTR sequence blocking miR‐1184 binding sites were cloned to build reporter plasmids as well as mutant vectors. It was detected that miR‐1184 mimic and reporter plasmids cotransfection strongly decreased luciferase activity. On the contrary, miR‐1184 mimic cotransfection with mutated vectors did not showed any apparent effects on luciferase activity. These data thus strongly indicate that IGFBP2 is a direct miR‐1184 target (Figure 3I,J).

### 3.4 circVANGL1 functions as a miR‐1184 sponge

Our analyses advised that miR‐1184 was the candidate circVANGL1 target. Dual luciferase reporter assays were therefore conducted in which mutated and wild‐type sequences from circVANGL1 were cloned to construct mutant vectors and reporter plasmids. We verified that miR‐1184 mimic and the reporter plasmid containing wild‐type circVANGL1 cotransfection strongly decreased reporter luciferase activity. On the contrary, miR‐1184 mimic and a mutant circVANGL1 vector containing mutated binding sites for miR‐1184 cotransfection showed no apparent effects regarding luciferase activity. The findings indicate that miR‐1184 is a direct circVANGL1 target (Figure 4A,B). Quantitative reverse transcription PCR assays were then performed to show that miR‐1184 expression had no effect on circVANGL1 expression in SV‐HUC cells transfected with the miR‐1184 mimic (Figure 4C), but after transfection with the circVANGL1 overexpression vector, miR‐1184 levels in SV‐HUC cells were significantly decreased (Figure 4D).

**Figure 4:** Circular RNA VANGL1 (circVANGL1) acts as a sponge for miR‐1184. A, Binding sites of miR‐1184 in circVANGL1 were predicted. The mutated version of circVANGL1 is also shown. B, Relative luciferase activity was determined 48 h after transfection with miR‐1184 mimic/NC or with circVANGL1 wild type (WT)/Mutant (Mut) in HEK293T cells. Data are presented as means ± SD. ***P < .001 vs control. C, Quantitative reverse transcription PCR (qRT‐PCR) analysis of the effect of expressing circVANGL1 in UM‐UC‐3 cells after transfection with miR‐1184 mimics. GAPDH expression levels were detected as an endogenous control. D, qRT‐PCR analysis of the effect of expressing miR‐1184 in UM‐UC‐3 cells after transfection with a circVANGL1 overexpression vector. GAPDH expression levels were detected as an endogenous control. Data are presented as means ± SD. ***P < .001 vs control

To identify the interaction between circVANGL1 and miR‐1184 in the progression of BC, SV‐HUC cells were transfected with the circVANGL1 silencing vector or were treated with miR‐1184‐specific inhibitor. The results showed that circVANGL1 downregulation significantly increased miR‐1184 expression and that miR‐1184 inhibitor suppressed miR‐1184 expression (Figure 5A). Western blots showed that IGFBP2 expression decreased in UM‐UC‐3 cells after circVANGL1 was silenced, but was strongly enhanced after treatment with miR‐1184 inhibitor (Figure 5B,C). CCK8 assays demonstrated that the downregulation of miR‐1184 expression after silencing circVANGL1 significantly decreased the UM‐UC‐3 proliferation compared to control cells, while treatment with miR‐1184 inhibitor increased UM‐UC‐3 cell proliferations even after circVANGL1 was silenced (Figure 5D) Wound‐healing assays indicated that the upregulation of miR‐1184 after circVANGL1 silencing caused slower closure of scratch wounds comparing with the control group, but miR‐1184 inhibitor treatment promoted faster closing of scratch wounds (Figure 5E). Also, Transwell invasion and migration assays found that the invasive and migratory capacity of UM‐UC‐3 cells was diminished after increasing miR‐1184 expression with circVANGL1 silencing, but increasing IGFBP2 levels with miR‐1184 inhibitor treatment promoted migration and invasion by UM‐UC‐3 cells (Figure 5F‐H). These outcomes suggested that downregulating miR‐1184 effectively reversed BC cell migration, invasion and growth after circVANGL1 silencing.

**Figure 5:** Downregulation of miR‐1184 effectively reverses the inhibition of bladder cancer (BC) cell growth, migration and invasion after silencing circular RNA VANGL1 (circVANGL1) in vitro. UM‐UC‐3 cells were transfected with miR‐1184‐control, miR‐1184‐inhibitor, sicircVANGL1 or miR‐1184‐inhibitor + circVANGL1. A, Quantitative reverse transcription PCR (qRT‐PCR) detection shows the expression of miR‐1184 and circVANGL1. Data are presented as means ± SD. ***P < .001 vs control. ^###^ *P* < .001 vs small interfering RNA against circVANGL1 (sicircRNA). B, Western blot shows insulin‐like growth factor‐binding protein 2 expression. C, Relative protein levels were analyzed and data are presented as means ± SD. *P < .05, ***P < .001 vs control. ^###^ *P* < .001 vs sicircRNA. D, CCK8 assays were performed to assess cell proliferation. Data are presented as means ± SD. ***P < .001. E, Wound‐healing assays showed that downregulation of circVANGL1 resulted in slower closure of scratch wounds. Scale bars: 30 μm. F‐H, Cell migration and invasion were determined in UM‐UC‐3 cells using Transwell assays. Data are presented as means ± SD. ***P < .001 vs control. ^###^ *P* < .001 vs sicircRNA. Scale bars: 50 μm

### 3.5 Silencing circVANGL1 suppresses nude mice xenografts tumor formation

To assess whether silencing circVANGL1 exerts a tumor inhibitory effect in vivo, we established a xenograft mouse model by subcutaneously injecting equivalent amounts of UM‐UC‐3 cells (six cells per group). The data suggested that silencing circVANGL1 significantly suppressed tumor volume comparing with the wild‐type UM‐UC‐3 group (Figure 6A‐C). Quantitative reverse transcription PCR analysis further informed that miR‐1184 expression was increased in the circVANGL1‐silenced group (Figure 6D), while IGFBP2 expression was downregulated (Figure 6E). Western blot further confirmed that circVANGL1‐silenced decreased IGFBP2 expression in protein level (Figure 6E).

**Figure 6:** Silencing circular RNA VANGL1 (circVANGL1) suppresses tumor formation in nude mice xenografts. A, Representative image of nude mice injected with UM‐UC‐3 cells. B, Representative picture of tumor formation in xenografts of nude mice (n = 6). C, Summary of tumor volumes in mice measured every week. D and E, Quantitative reverse transcription PCR detection shows the expression of miR‐1184 (D) and insulin‐like growth factor‐binding protein 2 (IGFBP‐2) (E). Data are presented as means ± SD. ***P < .001 vs control. F, Western blot detection show the expression of IGFBP‐2

## 4 DISCUSSION

More confident evidence has verified that circRNAs function crucially in cancer development and progression.^22^, ^23^ Nevertheless, their functions in BC remain largely unclear. In current investigation, we validated that circVANGL1 expression increased in both BC patients and BC cell lines. Circular RNA VANGL1 downregulation suppressed cell invasion, migration and growth. The results also showed that silencing circVANGL1 suppressed IGFBP2 expression. Insulin‐like growth factor‐binding protein 2 is validated as a candidate cancer marker because it is a protein secreted that is already explored in the plasma. High levels of it have been repeatedly correlated with disease severity in cancer.^24^, ^25^ Circulating IGFBP2 has demonstrated as a candidate marker for predicting the cancer prognosis including that of gastric cancer.^26^ In lung cancer, overexpressed IGFBP2 enhances cell activity and chemoresistance by enhancing autophagy.^27^ However, while IGFBP2 is a candidate target with therapeutic mechanism in cancer,^28^ its role in the progression of BC is still unclear.

In addition, we found that miR‐1184 functions importantly in BC. miR‐1184 overexpression significantly suppressed cell invasion, migration and growth, and silencing circVANGL1 promoted miR‐1184 expression. We also found that circVANGL1 might be a miRNA sponge by interaction with miR‐1184 and suppressing its activation. miR‐1184 suppression reversed its inhibitory effect on cell invasion, growth and migration and after silencing circVANGL1. It thus appears that miR‐1184 is the downstream circVANGL1 action target.

The results revealed that miR‐1184 can interact with the IGFBP2 3′UTR and suppress IGFBP2 expression at the posttranscriptional level. Increased IGFBP2 expression reversed the miR‐1184 inhibitory effect on cell migration, invasion, and growth. Recent studies have demonstrated that miR‐204‐3p overexpression enriched glioma cell apoptosis by targeting IGFBP2,^29^ and that downregulating IGFBP2 suppressed glioma cell invasion and migration.^30^ Taken together with our study results, these results indicated an indispensable tumor‐suppressor mechanism for the miR‐1184/IGFBP2 pathway in BC.

In summary, our results found that circVANGL1 expression promoted oncogenesis by sponging miR‐1184, indicating that circVANGL1 might be a promising prognostic biomarker for BC. The novel circVANGL1/miR‐1184/IGFBP2 axis may thus provide an effective therapeutic target for fighting BC.

## CONFLICT OF INTEREST

None declared.

## AUTHOR CONTRIBUTIONS

BL and DL conceived the research and drafted the paper with feedbacks of all authors. DY, HQ, and ZF performed the experiments and analyzed the data. AX and SZ carried out experiments and revised the draft. All authors approved the final version of the draft.
